The article "The role of NF-κB and miRNA in oral cancer and cancer stem cells with or without HPV16 infection" was retracted in 2020. Reasons: manipulated images; duplicated images; concerns about the data; concerns about the images.

# The role of NF-κB and miRNA in oral cancer and cancer stem cells with or without HPV16 infection

**DOI:** 10.1371/journal.pone.0205518

**Published:** 2018-10-29

**Authors:** Nasreen Bano, Manisha Yadav, Dheeraj Mohania, Bhudev C. Das

**Affiliations:** 1 Dr. B.R. Ambedker Centre for Biomedical Research, University of Delhi, New Delhi, India; 2 Sir Ganga Ram Hospital (S.G.R.H.) Rajinder Nagar, New Delhi, India; 3 Stem Cell & Cancer Research Lab, Amity Institute of Molecular Medicine & Stem Cell Research (AIMMSCR), Amity University, Uttar Pradesh, Noida, India; University of South Alabama Mitchell Cancer Institute, UNITED STATES

## Abstract

A small subpopulation of cancer stem-like cells (CSCs) present in almost all tumors is responsible for drug resistance and tumor recurrence. The role of NF-kB and miRNA in close association with essential risk factors, tobacco, alcohol and high risk HPV infection during oral carcinogenesis and its prognosis is not well understood. We have isolated cancer stem like SP cells from both HPV+/-ve oral squamous cell carcinoma (OSCC) cell lines and primary tumors, which formed orospheres, expressed stemness markers Oct4, Sox-2, CD133 and CD117. These cells showed differentially upregulated expression of NF-kB proteins and selective overexpression of viral oncogenes E6/E7 only in HPV16+ve cells which formed higher number of orospheres, overexpressed c-Rel and selectively activated p65 that heterodimerized with p50 to show higher DNA binding activity. Further, selective over expression of miR-21 and miR-155 and downregulation of miR-34a were demonstrated by HPV+ve CSCs which overexpress HPV16 oncogene E6 that is responsible for the maintenance of stemness. While, HPV-ve CSCs show exclusively p50 homodimeriztion, poor differentiation and worst prognosis, HPV infection induced participation of p65 along with deregulated expression of specific miRNAs led to well differentiation of tumors and better prognosis.

## Introduction

Head and neck squamous cell carcinomas (HNSCCs) are the most common cancers in developing countries, especially in southeast Asia [1]. Despite advances in treatment that includes mainly surgery and chemo-radiotherapy, the 5-year survival has remained approximately 50% for the last 10 years. Failure to treatment and reduced survival include late stage diagnosis, resistance to therapy, local recurrence and distant metastasis [2, 3].

Oral squamous cell carcinoma (OSCC) is one of the most predominant sub-type of HNSCC highly prevalent in India [4]. Although majority of the OSCCs are associated with smoking and alcohol consumption, a significant proportion of oral cancer has been demonstrated to contain high risk human papilloma virus (HR-HPV) infection [5]. The HR- HPV infected OSCCs and other HNSCCs show distinct characteristics when compared to their HPV negative counterparts, HPV-positive oral cancer patients show much better prognosis as compared to HPV-negative HNSCCs, with better response to chemotherapy, radiation, and surgery [6–9]. These patients also show improved immune response [10] and lower likelihood of metastasis with well differentiated tumors [6, 11] than the HPV-negative patients who show poorly differentiated tumors [11] and worst prognosis [6, 12]. It has been further shown that selective participation of NF-kB/p65 in HPV+ve tumors induces well differentiation and good prognosis [6].

NF-κB is a proinflammatory transcription factor that plays a pivotal role in initiation and progression of many cancers including HNSCCs and OSCCs [6, 13–15]. It consists of 5 distinct subunits that belong to the Rel family: RelA (p65/RelA), RelB, cRel (Rel), p50/p105 (NF-κB1) and p52/p100 (NF-κB2) which share an N-terminal Rel homology domain (RHD) responsible for DNA binding and homo- and heterodimerization. NF-κB normally remains in an inactive form in the cytoplasm through binding with inhibitory proteins IkBs, most notably IkBα [16] but upon activation in response to a variety of stimuli such as cytokines, lipopolysaccharide, stress signals, bacterial or viral infection, growth factors, chemotherapeutic agents, it gets translocated on to the nucleus and promotes expression of over hundred critical downstream target genes which are involved in variety of cellular functions including cell proliferation, apoptosis, cell migration and angiogenesis [17]. Also, HR- HPV 16 has also been shown to modulate NF-κB activation and expression in different cancers including OSCCs [6, 18, 19].

Apart from the HPV and NF-κB, a growing body of evidences indicate a critical role of small non-coding RNAs as microRNAs, the master regulators of transcription, in the initiation and progression of variety of human cancers including oral cancer [20–23]. The functional interaction between miRNAs and NF-κB and their signaling cascades are critical for tumor development and malignant progression. Several miRNAs are also shown to be differentially overexpressed in HPV-positive HNSCCs as compared to HPV negative HNSCC cells [24]. Also, various studies showed that miRNA expression pattern is affected by HPV status in human OSCCs [25, 26].

A large number of studies have delineated and validated an important pathophysiological role of a small subpopulation of cancer stem cells (CSCs) in long-term sustenance of cancer [27]. CSCs are the major source of drug resistance as they survive chemo-radiotherapy by exclusion of cytotoxic drugs using ABC transporter transmembrane proteins, reconstitute the tumor, and subsequently leading to tumor recurrence [28, 29]. Thus, CSCs drive the perpetuity of the disease making them difficult targets for standard cancer therapies [29]. CSCs as in normal stem cells maintain self-renewal and pluripotency [30]. Infection of HPV in the basal layer of epithelial cells interferes with differentiation and causes alteration in pluripotency genes [31]. It has also been shown that the NF-κB pathway is activated preferentially in the CSC of various malignancies leading to its constitutive activation, the functional implications of which appear to be self-renewal and maintenance of the CSC population [30].

The contribution of NF-κB and miRNA in oral carcinogenesis and their role in maintenance of oral cancer stem cells with or without HPV infection is unknown. We have therefore investigated the role of NF-κB and its family proteins along with selected miRNAs in SP (sphere forming stem cells), Non SP and parental OSCC cells derivedfrom cell lines as well as fresh tumor tissues to understand the role of NF-κB and miRNAs in presence or absence of HPV infection for tumorogenic progression and prognosis of oral cancer.

## Results

### HPV diagnosis and pathological classification of tumors

Out of 12 fresh oral cancer biopsy collected, 5 were HPV 16 positive and 7 were negative for any HPV. The differentiation status of the tumors and their histopathological diagnosis was provided from the pathology department of Sir Ganga Ram Hospital, New Delhi, India, where a part of tumor biopsies was retained for histopathological diagnosis. Of 12 tumor tissue biopsies 4 (80%) out of 5 HPV positive tumors were well differentiated and only one (20%) was moderately differentiated tumors while of 7 HPV-ve tumors, only 1 (14%) was well differentiated, 2 (28%) were moderately differentiated and 4 (57%) were poorly differentiated tumors. Out of 5 HPV positive tumors, 3 (60%) belonged to stage I-II while 2 (40%) belonged to stage III-IV. Of 7 HPV-ve tumors, 3 (42%) were of stage I-II and 4 (57%) were in stage III-IV. The details are presented in Table 1.

**Table 1:** HPV diagnosis, histopathological stages and grades of fresh oral cancer biopsies.

Characteristics	Differentiation/Stage	No. of Cases	HPV16+ve	HPV-ve
**Cancerous (n = 12)**	**WDSCC**	**5**	**4**	**1**
	**MDSCC**	**3**	**1**	**2**
	**PDSCC**	**4**	**-**	**4**
**TNM Staging**	**Stage I-II**	**6**	**3**	**3**
	**Stage III-IV**	**6**	**2**	**4**

**Abbreviations:** WDSCC; well-differentiated squamous cell carcinoma, MDSCC; moderately-differentiated squamous cell carcinoma, PDSCC; poorly-differentiated squamous cell carcinoma.

### Side population contains cancer stem like cells in HPV+ve and HPV-ve OSCC cell lines and fresh tumor primary culture

Flow cytometric analysis was performed both in HPV16 positive (UD-SCC2) and HPV negative (UPCI:SCC131 and UPCI:SCC84) OSCC cell lines and in HPV+ve/HPV-ve oral tumor primary culture for isolation of side population as CSCs on the basis of chemoresistance property of CSCs using Hoechst 33342 dye exclusion and its inhibitor verapamil. Cell sorting was performed after excluding dead cells and cellular debris based on scatter signals and propidium iodide (PI) fluorescence. The gated portion showed the SP cells that were Hoechst 33342 negative/dim and remaining cell population present outside the gated area indicated the Non-side population (NSP) cells that were Hoechst 33342 positive/bright. SP cells occupied 1.4%, 1.0% and 1.2% of the total cells in UD-SCC2 (HPV16+ve) (Fig 1A-i), UPCI:SCC131 (HPV-ve) (Fig 1A-ii) and UPCI:SCC84 (HPV-ve) (Fig 1A-iii) cell lines respectively whereas 2.1% and 1.4% of the total cells in HPV+ve (Fig 1B-i) and HPV-ve oral tumor primary culture (Fig 1B-ii). When pre-incubated with its inhibitor verapamil for 30 min, the percentage of SP cells shrank to 0.6%, 0.4% and 0.00% of total cells respectively in UD-SCC2, UPCI:SCC131 and UPCI:SCC84 while 0.1% and 0.5% in HPV+/-ve oral primary culture (Fig 1(A) and 1(B), S1 and S2 Figs).

**Fig 1:** Flow cytometric (FACS) analysis of SP cells in OSCC cell lines and OSCC biopsy. **A.** Flow cytometric analysis of side population (SP) in **(i)** UD-SCC2 (HPV16+ve), **(ii)** UPCI: SCC131 (HPV-ve) and (i**ii)** UPCI:SCC84 (HPV-ve) OSCC cell lines and **B(i)** oral tumor biopsy (HPV16+ve) **(ii)** and oral tumor biopsy (HPV-ve). OSCC cells were stained with Hoechst 33342 dye alone or in the presence of verapamil and analysed by flow cytometry measuring Hoechst blue vs Hoechst red fluorescence. The SP cells was gated and represented as a percentage of the whole viable cell population following propidium iodide exclusion.

### Oral cancer stem like cells form anchorage-independent, self-renewing orospheres

Single cell suspensions of sorted SP cells from three OSCC cell lines and oral cancer primary cultures were seeded at a density of 1X10^4^ cells on 6- well plates precoated with 1.2% Poly-HEMA in serum free DMEM-F12 medium. Cells grew as non-adherent, three-dimensional sphere clusters, called orospheres. Figs 2A(i)–2A(iii) and 3A(i) and 3A(ii) showed anchorage-independent spheres formed by OSCC SP cells sorted from above three cell lines and OSCC primary culture respectively. However, high number of loose sphere formation was observed in HPV+ve UD-SCC2 cells when compared to both HPV+ve/-ve cells and OSCC primary culture which formed compact spheres. HPV+ve UD-SCC2-SP cells formed a high degree of spheres which were distinctly larger than those observed in UPCI:SCC131-SP and UPCI:SCC84-SP cells (Fig 2B-i) with SFE (UD-SCC2-SFE,0.32%; UPCI:SCC131-SFE-,0.23%; UPCI:SCC84, 0.21%). Similar pattern of sphere forming efficiency was observed in OSCC+ve primary culture with comparatively high sphere forming efficiency (SFE) of 0.36% to that of 0.32% in OSCC HPV-ve specimens (Fig 3B-i). After 7 to 10 days, when the spheres grew to 70 to 100 μm in diameter, they were passaged and the single cell culture from these spheres was able to propagate to form new spheres again. Secondary and tertiary sphere formation was also observed in all three cell lines indicating their self-renewal capability in vitro. In contrast, we did not observe any spheroid formation from NSP cells, which either died or propagated very slowly but could not form visual spheres.

**Fig 2:** Functional characterization of SP cells present in OSCC cell lines. **A (i-iii).** Assessment of orosphere forming ability of SP cells. Representative photomicrograph of orosphere formation with sorted SP and Non-SP cells in low adherence defined Serum free media (DSFM) in (i) UD-SCC2, (ii) UPCI:SCC131 and (iii) UPCI:SCC84 (magnification 100X). **B (i).** Spheres with 0.75 mm diameter were counted after 10 days. The percentage of sphere forming cells was calculated by dividing the number of orospheres by the number of cells seeded in (i) OSCC cell lines. The experiments were performed at least three times and data are presented here as mean ± standard errors. UD-SCC2-SFE,0.32%; UPCI:SCC131-SFE,0.23%; UPCI:SCC84-SFE,0.21%, *P < 0.05 versus NSP cultures.

**Fig 3:** Functional characterization of SP cells present in OSCC tumor biopsies. **A(i-ii).** Assessment of orosphere forming ability of SP cells. Representative photomicrograph of orosphere formation with sorted SP and Non-SP cells in low adherence defined Serum free media (DSFM) in (i) oral tumor biopsy (HPV16+ve) and (ii) oral tumor biopsy (HPV-ve) (magnification 100X). **B (i).** Spheres with 0.75 mm diameter were counted after 10 days. The percentage of sphere forming cells was calculated by dividing the number of orospheres by the number of cells seeded in (i) OSCC biopsy. The experiments were performed at least three times and data are presented here as mean ± standard errors. OSCC biopsy (HPV+ve)-SFE,0.36%; OSCC biopsy (HPV-ve) -SFE,0.31%. *P < 0.05 versus NSP cultures.

### Oral cancer stem cells express CSC specific stemness markers

We next examined CSC marker expression in orospheres and compared with the expression levels in parental cells of HPV+ve and HPV-ve OSCC cell lines. The identification and characterization of cancer stem cell was done using markers CD133 and CD117 (c-kit). Inspite of limitations in using CD133 and CD117 as CSC marker, a large number of studies have used these markers for CSC identification and characterization. CD133 positive cells were found to be 21.19%, 12.32%, 57.51% for UPCI:SCC131, UPCI:SCC84 and UD-SCC2 SP cells respectively. CD117 positive cells were 13.52%, 11.95% and 64.48% for UPCI:SCC131, UPCI:SCC84 and UD-SCC2 SP cells respectively as compared to respective parental cells (Fig 4A and S3 Fig). These results suggest that sphere-forming SP cells, under stem cell-selective conditions, are enriched for CD133 and CD117 expressions.

**Fig 4:** Characterization of SP cells as cancer stem cells and expression of HPV16 E6 and E7 oncoprotein. **A.** Flow cytometric characterization identified SP cells as Cancer stem cell in (i) UD-SCC2, (HPV16+ve), (ii) UPCI:SCC131 and (iii) UPCI: SCC 084 (HPV-ve) cell lines using CD133 and CD117 cancer stem cell markers. Sphere-forming cells or SP cells and monolayer cells or parental cells were stained with CD117 and CD133 conjugated primary antibodies and subjected to flow cytometry. Red line corresponds to sphere-forming cells, black line to monolayer cells or parental cells as negative controls and green line to isotype control. Isotype matched mouse immunoglobulins served as controls**. (iv)** Bar graphs adjacent to histograms in each panel show Mean Fluorescent Intensity (MFI) of the peak at the higher fluorescence in the figure. Data from one of three independent experiments are shown (n = 3). The star above the bars represents the P value. The results were analyzed by one way ANOVA followed by Tukey’s post hoc multiple comparison test. * = P ≤ 0.05; ** = P ≤ 0.01; *** = P ≤ 0.001 and **** = P ≤ 0.0001. **B. OSCC express CSC markers: (i)** Western blot analysis of cancer stem cell markers from protein extract of sorted SP, NSP and parental cells from UD-SCC2 HPV16+ve, UPCI:SCC131 (HPV-ve)and UPCI:SCC84 (HPV-ve) cells. A total of 25 μg protein extracts each from SP, NSP and parental cells were separated on a 10% SDS-PAGE, electrotransferred on PVDF membrane and probed. To confirm equal protein loading, the membranes were reprobed for β-actin expression. **(ii)** The relative normalized fold change in the protein is expressed as the mean ±SD of three independent experiments. ***P value <0.*001*, **P value <0.*01*, *P value <0.*05* for UD-SCC2 HPV16+ve, UPCI:SCC131 (HPV-ve)and UPCI:SCC84 (HPV-ve) cells. **C (i-ii).** Representative photograph of EtBr-stained 2% agarose gel showing qRT-PCR amplification of HPV16 oncoproteins E6 and E7 in cDNA prepared from HPV16+ve SP, NSP and parental UD SCC2 cells and tumor biopsies. β globin was used as input control for normalization. **i &ii (lower panel):** Aggregated mean (± S.D.) abundance ratios of the transcripts w.r.t. β globin in three independent experiments. *p value ≤ 0.05 versus control NSP cells. Parental cells cultured in adherent condition were used as reference.

### Enhanced expression of cancer stemness markers and related proteins in HPV16+ve oral cancer stem cells

Expression of Oct-4, Sox-2 and CD44 was studied by western blot for further characterization of sphere forming SP cells as cancer initiating cells as compared to parental and NSP cells in oral cancer cell lines. We observed significantly upregulated expression of Oct-4, Sox-2 and CD44 in orosphere forming SP cells of UD SCC2 (HPV16+) cells than that of UPCI:SCC131, UPCI:SCC084 HPV-ve SP cells when compared to corresponding Parental and NSP cells as revealed by western blot analysis (see Fig 4Bi–4Biii).

### SP cells that form orospheres overexpress HPVE6/E7

qRT-PCR analysis of cDNA derived from Parental, SP and NSP cells of HPV16+ve, UD SCC2 cell line and CSCs derived from patient biopsies demonstrated significantly an increased level of E6 and E7 expression when compared with parental and NSP cells. SP cells characteristically overexpressed E6 and E7 transcripts (Fig 4Ci and 4Cii).

### Differential overexpression of specific NF-κB family proteins in oral cancer stem cells

Western blotting experiments were performed to study the expressions pattern of all five NF-κB family proteins, e.g., p50, p65, p52, c-Rel and RelB in Parental, NSP and SP cells of UPCI:SCC131 (HPV-ve), UPCI:SCC84 (HPV-ve) and UD-SCC2 (HPV+ve) cells. All three cell lines showed significantly a higher expression of all five NF-κB proteins, p65 (p = 0.0001), p50 (p = 0.0001), p52 (p = 0.0001), c-Rel (p = 0.0001) and Rel-B (p = 0.0001) in their SP cells as compared to their respective NSP and parental cells (Fig 5A and 5B). However, on observing expression of SP cells between HPV+ve and HPV-ve cells, we observed a significantly higher expression of p65 (p = 0.0001) and p50 (p = 0.0001) in HPV+ve cell line. Also, remarkably a very high level of expression of c-Rel (p = 0.0001) was found only in HPV+ve SP cells (Fig 5A and 5B) while p52 and Rel-B showed minor difference. No significant differential expression pattern was observed among NSP and parental cells of all three cell lines.

**Fig 5:** Differential expression pattern of NF-κB family proteins in OSCC cell lines. **A.** Western blot analysis of NF-κB family proteins in cellular protein extracted from sorted SP, NSP and parental cells from (i)UD-SCC2 HPV16+, (ii) UPCI:SCC131 and (iii) UPCI:SCC84 cell line. A total of 25 μg protein extracts each from SP, NSP and parental cells were separated on a 10% SDS-PAGE, electrotransferred on PVDF membrane and probed for NF-κB family proteins p65, p50, p52, c-Rel and Rel-B. To confirm equal protein loading, the membranes were reprobed for β-actin expression. The relative normalized fold change in the protein is expressed as the mean ±SD of three independent experiments. **B.** Bar diagram showing NF-κB family proteins expression between SP cells, NSP cells and Parental cells from (i) UD-SCC2 HPV16+, (ii) UPCI:SCC131 and (iii) UPCI:SCC84 cell lines. ***P value <0.*001*, **P value <0.*01*, *P value <0.*05*.

Similarly, SP cells from both HPV16+ve and HPV-ve tumor biopsies showed strong expression of all NF-κB family proteins, i.e. p50 (0.001), p52 (0.001), p65 (0.001), c-Rel (0.001), and RelB (0.001) with respect to their NSP and parental cells (Fig 6A and 6B). However, upon observing impact of HPV among SP cells of HPV+ve and HPV-ve biopsies, a slightly higher expression of p50 was observed mainly in HPV-ve cases as compared to HPV16+ve OSCCs that overexpressed specifically p65 and p52 proteins. Higher expression of c-Rel is also observed in HPV+ve clinical specimen’s SP cells, similar to UD-SCC2 (HPV16+) cells. While Rel-B showed minor difference among HPV+ve and HPV-ve OSCC cases, no significant differential expression was observed among NSP and parental cells of HPV+ve and HPV-ve OSCC cases. These data very well corroborate the results of bandshift assays of OSCC cell lines.

**Fig 6:** Differential expression pattern of NF-κB family proteins in OSCC biopsies. **A.** Western blot analysis of NF-κB family proteins in cellular protein extracted from sorted SP, NSP and parental cells from (i) HPV+ve OSCC biopsies and (ii) HPV-ve OSCC biopsies. A total of 25 μg protein extracts each from SP, NSP and parental cells were separated on a 10% SDS-PAGE, electrotransferred on PVDF membrane and probed for NF-κB family proteins p65, p50, p52, c-Rel and Rel-B. To confirm equal protein loading, the membranes were reprobed for β-actin expression. The relative normalized fold change in the protein is expressed as the mean ±SD of three independent experiments. **B.** Bar diagram showing NF-κB family proteins expression between SP cells, NSP cells and Parental cells from (i) HPV+ve OSCC biopsies and (ii) HPV-ve OSCC biopsies. ***P value <0.*001*, **P value <0.*01*, *P value <0.*05*.

### Preferential heterodimerization of p50 with p65 that formed functional NF-κB complex only in HPV+ve OCSCs

To dissect the composition of functional NF-κB complex formation in presence and absence of HPV in parental, NSP and SP cells of oral cancer cells, gel supershift assays were performed using specific antibodies raised against all five NF-κB family members (p50, p52, p65, c-Rel and RelB). As the results of both HPV-ve cell lines are similar in all other experiments, we have chosen only one of the HPV-ve cell lines i.e. UPCI:SCC84 for performing EMSA. The results demonstrated a slightly lower DNA binding of NF-κB in HPV16 infected cells than HPV negative cells (Fig 7A-i). On observing binding of NF-κB in all sets of OSCC cells i.e parental, NSP and SP, similar lower DNA binding activity of NF-κB has been found in HPV16 positive cells (Fig 7A-ii). However, a difference was also observed in binding activity in SP cells that show higher binding as compared to their parental and NSP counterparts both in HPV+ve and HPV-ve cells (Fig 7A-ii and S4 Fig). For checking NF-κB binding specificity, a competition assay has been done using Oct-1(as an internal control) in different OSCC cells using Oct-1 consensus sequence with 100 fold molar excess of homologous NF-κB and a heterologous Oct-1 cold probe (Fig 7Bi and 7Bii).

**Fig 7:** Effect of HPV16 infection on the constitutive activity of NF-κB and its composition in oral cancer stem cells. **A.** Constitutive activation and DNA binding activity of NF-κB in HPV+ve and HPV-ve oral cancer cells. EMSA showing DNA binding activity of NF-κB in nuclear extracts (10μg) of (i)HPV+ve and HPV-ve OSCC cells, (ii) in different sets of parental, NSP and SP cells of OSCC cell lines in both HPV+ve and HPV-ve cells using Cγ3- labeled oligonucleotide harboring an NF-κB consensus sequence. Fold change in the band intensities of NF-κB are indicated in each lane. The intensities of shifted bands quantified in densitometric analysis. **B.** EMSA showing binding specificity using nuclear extracts from OSCC cells, with a Cγ3-labelled oligonucleotide harboring an Oct-1 and NF-κB (right side) consensus sequence. (i) Oct-1 probe that showed consistent DNA binding in different sets of OSCC cells. (ii) Binding specificity was evidenced by pre-incubation with a 100 fold molar addition of the homologous unlabeled NF-κB oligonucleotide in comparison with competition experiments using a heterologous consensus sequence of the Oct-1 transcription factor. The positions of the specific retarded bands are indicated. **C.** Supershift assay showing altered composition of functional NF-κB complex in HPV+ve and HPV−ve OSCC cells. Nuclear extracts (10 μg) prepared from (i) SP, parental and NSP cells from oral cancer cell line UPCI:SCC84 (HPV-ve), (ii) SP, parental and NSP cells from UD-SCC2 (HPV+ve) oral cancer cell line as well as respective nuclear extracts were incubated with specific antibodies (2 μg each) against each of p65, p50, p52, c-Rel, RelB and assayed for NF-κB binding activity by band supershift asssay as described in Methods and band intensities quantified are indicated. The arrowhead indicates the super-shifted bands.

The results of gel supershift assay revealed p50 as the major DNA binding partner involved in the formation of p50:p50 homodimer as the functional NF-κB complex in HPV negative oral cancer cells whereas HPV16 positive cells showed selective participation of p65 along with p50 (Fig 7C-i). No shift was observed for other NF-κB family proteins in both HPV positive and HPV negative oral cancer cells. As such in HPV negative parental, NSP and SP cells, functional NF-κB complex was formed by mainly p50-p50 homodimer (Fig 7C-i) while HPV16 infection induced selective participation of p65 in UD-SCC2 cells (Fig 7C-ii).

Also, SP cells in the absence of HPV infection showed higher (~ 85%) supershift of p50 in functional NF-κB complex formation as compared to that of parental and NSP cells which showed lesser involvement (~ 40–60%) in their p50-p50 homodimer formation while no other NF-κB family proteins are involved in functional dimer formation (Fig 7C-i). Interestingly, HPV16 positive SP cells (UD-SCC2) showed very strong involvement of p65 with p50 (Fig 7C-ii) with about 90% supershift of p65 subunit while only 40% of supershift of p50 was found (Fig 7C). Together, these results indicate a strong DNA binding activity of NF-κB and selective participation of p65 in the formation of functional NF-κB complex in oral cancer stem like cells in the presence of HPV while in absence of HPV, p50-p50 homodimer formation was always observed.

### Differential expression of selected miRNAs in OSCC stem cells

The small non-coding RNAs, the miRNAs which are considered as master regulator of post transcriptional gene expression, can function as oncogenes or tumor suppressor genes and play a pivotal role in tumor initiation and progression. In the present study, we looked for expression pattern of three selected miRNAs, two oncogenic, miRNAs, miR-21 miR-155 and one tumor suppressor miRNA, miR-34a which are frequently associated and are known to play critical role in OSCC. The expression of these three miRs was determined in HPV positive and HPV negative SP, NSP and parental cells. Out of three miRs, miR-21 and miR-155 were consistently upregulated whereas miR-34a was regularly downregulated in SP cells of all three OSCC cell lines as compared to that of their respective parental counterparts. The fold change expression level in SP cells of HPV+veUD-SCC2, HPV-ve UPCI:SCC131 and UPCI:SCC84 cell lines for miR-21 were 1.83, 1.29, 1.13 whereas for miR155 were 1.85, 1.20, 1.44 and that of miR-34a was 0.066, 0.27and 0.31 respectively which were significantly different from those of respective parental cells (see Table 2 and Fig 8i–8iii). Whereas in NSP cells, all three miRNAs screened were consistently downregulated as compared to that of their respective parental cells except higher miR-155 expression in HPV positive NSP cells. The fold change expression level in NSP cells of HPV+veUD-SCC2, HPV-ve UPCI:SCC131 and UPCI:SCC84 cell lines for miR-21 were 0.89, 0.72,0.59 whereas for miR-155 were 1.2, 0.862, 0.87 and that of miR-34a were 0.39, 0.71, 0.27 respectively (see Table 2 and Fig 8i–8iii) which are also significantly different from those of respective parental cells. Overall, expression of these three miRNAs changed in CSCs (SP) when compared to that of non-CSCs (NSP) and parental cells, and increased in relation to HPV infection (S5 Fig and S1 Table).

**Fig 8:** Relative expression level of selected miRNAs in SP, NSP and their parental controls from UD-SCC2 (HPV16+ve), UPCI:SCC131 (HPV-ve) and UPCI: SCC 084 (HPV-ve) cells. **(i-iii).** The relative expression level of (i) miR-21, (ii) miR-34a and (iii) miR-155 in SP, NSP and their parental controls from HPV+ve (UD-SCC2), HPV-ve (UPCI:SCC131) and HPV-ve (UPCI:SCC84) cell lines. SP cells show higher expression of miR-21 and miR-155 while it showed downregulation of miR-34a expression.***P value <0.*001*, **P value <0.*01*, *P value <0.*05*. *Parental versus corresponding SP*.

**Table 2:** Relative miRNA expression level in OSCC in SP and NSP cells with parental cells as their respective controls for HPV+ve UD-SCC2, HPV-ve UPCI: SCC131 and UPCI:SCC84 cell lines.

miRNA types	SP cells (CSCs)									
	UD-SCC2			UPCI:SCC131				UPCI:SCC84		
	FC±SE	P value	Regulation	FC±SE	P value	Regulation		FC±SE	P value	Regulation
**miR- 21**	**1.836±0.03**	0.001*	**Up**	**1.29±0.03**	0.001*	**Up**		**1.13±0.07**	0.01*	**Up**
**miR-34a**	**0.066±0.013**	0.001*	**Down**	**0.27±0.02**	0.0001*	**Down**		**0.31±0.02**	0.001*	**Down**
**miR-155**	**1.85±0.04**	0.001*	**Up**	**1.20±0.04**	0.05*	**Up**		**1.44±0.15**	0.001*	**Up**
**NSP cells**										
**miR- 21**	**0.8935±0.05**	0.001*	**Down**	**0.724±0.038**	0.001*		**Down**	**0.59±0.03**	0.001*	**Down**
**miR-34a**	**0.39±0.09**	0.001*	**Down**	**0.71±0.0.15**	0.001*		**Down**	**0.27±0.02**	0.001*	**Down**
**miR-155**	**1.2±0.103**	0.05*	**Up**	**0.862±0.107**	**P>0.05**		**Down**	**0.87±0.09**	**p>0.05**	**Down**

**Abbreviations:** SP: Side population; NSP: Non- Side population; FC: Fold change; S.E: Standard Error.

*Significant

## Discussion

The conventional cancer therapeutic strategies are mainly focussed on tumor regression by targeting to kill only the bulk of the differentiated tumor cells but they always spare a small population of CSCs that possess the capacity of self-renewal and ability to drive continued expansion of tumor later leading to relapse of the disease [31]. Since aberrant activation and overexpression of the proinflammatory transcription factor, NF-κB plays a key role in regulating wide variety of cellular processes including cell differentiation, apoptosis, transformation and signal transduction pathways, specifically during progression and metastasis of several cancers including oral cancer, it is important to unpave the role of NF-κB proteins. It has been shown that the NF-κB pathway is activated preferentially in cancer and CSCs of diverse malignancies, including leukemia, glioblastoma, prostate, ovary, breast, pancreatic and colon cancer and its activation is known to induce radio- and chemotherapy resistance [32–38]. In addition, miRNAs are yet another important regulatory molecule involved during carcinogenesis; they themselves can act as oncogenes or tumor suppressor genes and functionally interact with NF-κB and other molecules. This prompted us to examine interaction between NF-κB, miRNA and HPV during pathogenesis and prognosis of oral cancer. We report here the presence of oral cancer stem like cells (OCSCs) which show self renewal property and tumorosphere formation ability in both HPV+ve (UD-SCC2) and HPV-ve cells (UPCI: SCC131 and UPCI: SCC84) including HPV+ve/HPV-ve primary oral tumor specimens. Although identification and isolation of cancer stem like cells from oral cancer cell lines has been reported previously [39] but no correlation has been made with HR-HPV16, present in substantial proportion of OSCCs as well as with NF-κB or miRNA which play a critical role during progression and prognosis of oral cancer. The present study defines the role of specific NF-kB family proteins and miRNA and their interactive contribution in differential pathogenesis, prognosis and stemness in presence or absence of HPV infection.

Of various approaches, the identification and isolation of CSCs was done with ABCG2 receptor expression by measuring the active efflux of its fluorescence substrate, Hoechst 33342, in the presence/absence of its inhibitor verapamil. We observed verapamil-sensitive SP population in all three cell lines alongwith primary oral cancer specimens. Significantly a higher proportion of SP cells were always detected in HPV+ve (UD-SCC2) cell line as well as in HPV+ve oral tumor specimens. This is in concordance with the earlier reports [40, 41]. Furthermore, we observed that both HPV+ve and HPV-ve SP cells formed orospheres, a hallmark feature of stemness, self–renewal property and tumorigenicity but distinctly a higher number of loose spheres were formed by HPV+ve SP cells. Our observation of a higher proportion of CSCs and higher sphere-forming ability may be attributed to the presence of HPV16 that show an increased expression of its oncoprotein E6. Our hypothesis gains support from the observations of other studies in which high-risk HPV16 significantly increased the tumorosphere forming ability [42] and elevated CSC population, [43]. HPV16 E6 oncoprotein has been credited for the increased CSC production, tumorosphere formation and tumorigenesis through dysregulation of p53 and it is suggested that viral oncogenes can induce stem cell–like phenotype in human keratinocytes/epithelial cells by interfering with their differentiation [40, 44]. Recently, it has also been demonstrated in cervical cancer that HPV 16 oncoptotein E6 selectively overexpresses in cervical cancer stem like cells and participates in maintenance of stem cell phenotype and stemness through upreulation of Hes1 [40].

Apart from Hoechst–based SP analysis, we further characterized CSCs by epithelial cancer stem cell markers CD133 and CD117 which are often used to characterize CSCs in various cancers including head and neck and oral cancer [45, 46]. The expression of these markers was significantly higher in CSCs that were positive for HPV16 than the HPV-ve SP cells. CD133 expression is known to be associated with activation of c-Src and required for maintenance of CSC phenotype through EMT modulation in head and neck cancer [47] CD133 rich subpopulations of orospheres with self-renewal capacity are exclusively tumorigenic [45, 48]. The HPV+ve orospheres show a higher expression of Sox2 and Oct4 than that of HPV-ve SP cells whereas very little or basal expression was seen in parental and NSP cells of both HPV+ve/ HPV-ve cells. Similarly CD44 expression was found to be significantly higher in HPV+ve SP cells. These observations further strengthen our findings that HPV infection is not only essential for malignant progression but also required for maintenance of stemness properties of CSCs.

Deregulation of p53 and Rb through interaction with HPV oncogene E6 and E7 respectively leads to increased CSC production and it is an important cellular pathway in maintaining stemness [49, 50]. It is interesting to note higher expression of E6 and E7 specifically in undifferentiated SP cells while relatively lower level was observed in differentiated NSP cells. This finding well correlates with our hypothesis of attribution of higher proportion of CSCs and enhanced sphere-forming ability to HPV. Our finding of higher expression of HPV E6/E7 oncogenes in CSCs was also corroborates our recent report by Tyagi et al, (2016) which show higher expression of E6 specifically in cervical cancer stem cells that has been shown to control stemness and self-renewal through upregulation of HES1 as CSCs are more permissive to HPV infection. Also, Lee and colleagues [42] has shown in HPV-ve OSCC cells that after introduction of whole genome of HPV into these HPV-ve cells, it increased tumorigenicity in OSCC by enhancing the stemness through downregulation of specific miRNA. Also it is consistent with reports linking inactivation/loss/blocking of p53 as an essential mechanism to enhance the CSC population in HPV16-positive OPSCC [43], pluripotent stem cells [51–53] and mammary stem cells [54].

NF-κB signaling is known to regulate cell proliferation, differentiation, apoptosis, and stemness [33] and plays an important role in oral carcinogenesis [6]. Our bandshift and immunoblotting results demonstrate higher DNA binding and differential overexpression of NF-κB family proteins in SP cells from all three cell lines but their expression and binding were certainly higher in HPV+ve SP cells (UD-SCC2). There is a selective participation of p65 with p50 to form functional NF-κB complex only in HPV+ve cells. These findings very well corroborate with the immunoblotting results from freshly collected oral cancer specimens. It gains strong support from our earlier findings [6] which showed for the first time that p65 participation in the presence of HPV induced well differentiated tumors and better prognosis [6]. However, the mechanism(s) underlying these observations was unclear. Our observation of regular involvement and higher expression of p65 well correlate with other findings where NF-κB inhibition in CSCs reduced self-renewal and stopped xenograft tumor growth [55]. It is intriguing that while HPV infection increased tumorosphere formation and stemnes of oral CSCs but at the same time HPV infection activates p65 which participates in transactivation leading to well differentiation of tumors leading to better prognosis when treated. An indispensable role of NF-kB/p65 in growth and differentiation during embryonic development and liver regeneration has been demonstrated in p65 knockout mice [56] and selective suppression of p65 in HEV infected pregnant women [57] leads severe liver degeneration, liver failure and death of both foetus and mother.

It is interesting to note that c-rel is highly overexpressed in HPV+ve SP cells derived from both UD-SCC2 cell line and HPV16+ve primary oral tumor specimens. Such overexpression or amplification and/or rearrangement of c-Rel gene has been often observed in many aggressive solid tumors as well as hematopoietic malignancies [6, 58, 59]. Interestingly enough, our group has recently shown a significant higher expression of c-Rel in HPV-ve tongue cancer instead of HPV+ve tumors which has been observed in oral cancer. This is intriguing but it indicate that expression of cancer associated genes may differ from cancer to cancer along with their grades/stages [60].

It is also known to control epidermal development and homeostasis in embryonic and adult skin [61]. Activation of c-Rel has been shown to induce expression of NF-κB target genes such as cyclin D1, c-Myc, and Bcl-xL, which play pivotal role in tumor growth [62] including induction c-Jun and CDKs that promote cell proliferation and aggressive tumor phenotype [63–65]. Since cellular differentiation is frequently characterized by G1 arrest, consistent with this is the observation that c-rel can promote G1 arrest and increase p21/Cip1 expression in the transformed HPV positive HeLa cell line [66]. Also, p21/Cip1 has been shown to be over-expressed in the HPV infected laryngeal papillomas [67]. Earlier it was shown by us an over-expression of p21 in well-differentiated oral squamous cell carcinomas (WDSCCs) which showed better prognosis [6]. p21WAF1/CIP1 is a downstream mediator of p53 which mediates growth arrest by inhibiting the action of G1 cyclin-dependent kinases. As cancer stem like cells also show characteristic quiescence and remains in G1/Go phase with slow cell division and show overexpression of c-Rel which can affect cell cycle control and involved in the p21WAF1 and p53 mediated cell cycle regulation. These observations together indicate a critical role of HPV in altering composition of functional NF-κB complex and differential expression of NF-κB proteins in oral cancer stem like cells involved in the maintenance of their stemness and but at the same time facilitates better differentiation leading to good prognosis when treated. This is also true that though both HPV+ve and HPV-ve cells/tumors contain CSCs, selective activation of NF-kB/p65 in presence of HPV causes activation of immune response, enhance cell proliferation and better differentiation leading to good prognosis [6, 10, 11, 56].

Furthermore, we explored the role of three specific miRNAs which interacts with NF-κB during oral carcinogenesis. We observed higher expression of two oncogenic miRNAs; miR-155 and miR-21 in HPV+ve SP cells compared to HPV-ve SP cells (Fig 6-i & 6iii). It well correlates with recent reports which demonstrate that HPV infection affect miRNA expression pattern in human SCC [26, 68]. It is important to note that miR-155 is an NF-κB transactivational target and is involved in a negative feedback loop through downregulation of IKKs and other genes. Taken together, our observations are consistent with the recent studies which support a positive association between oncogenic miR-155/miR-21 upregulation and NF-κB activation; both contributing to oral carcinogenesis [69–71]. In contrast, the expression of miR-34a is significantly downregulated in both HPV+ve and HPV-ve SP cells, however this downregulation is more pronounced in HPV positive SP cells (Fig 8-ii). As miR-34a is transcriptionally regulated by p53, it controls the expression of a plethora of target proteins involved in cell cycle regulation, differentiation and apoptosis and inhibits cancer cell viability, stemness and metastasis. Our observations are consistent with Wang et al., (2009) who showed downregulation of miR34a in HPV infected cervical cancer [72]. Down-regulation of miR-34a can be attributed to the high-risk HPV E6 oncoprotein which mediates degradation of p53 [73, 74]. Consequently, miR-34a is also downregulated providing a growth advantage for HPV+ve CSCs.

On the basis of above results, we propose here a plausible model (Fig 9) that demonstrates the role of human papillomavirus oncogenes in modulating the function of NF-κB and miRNAs in oral cancer contributing towards its progression, metastasis and treatment outcome. HPV16 infection that appears to enhance the stem cell population, their stemness properties and orosphere formation ability of oral CSCs, but HPV also activates p65 that induced better differentiation. HPV also does this through functional interaction with NF-κB proteins by altering the composition of NF-κB p50/50 homodimer in favour of p50/p65 heterodimer. The selective participation of p65 and exclusive overexpression of c-Rel in HPV positive OSCCs facilitated well differentiation leading to better prognosis. In contrast, in absence of HPV there is no involvement of p65 in the functional NF-κB complex and no overexression of c-Rel leading to poorly differentiated, invasive and metastatic tumor that show worst prognosis. The interaction between activated NF-κB protein, their transactivation and HPV oncoproteins and overexpression of miR-155/miR-21 and miR-34a downregulation all appears to contribute towards well differentiation and better prognosis when treated. Yet HPV16 plays a crucial role in maintaining stemness of oral cancer stem like cells through up regulated expression of viral oncogenes (E6/E7) and its functional interaction with NF-κB proteins and specific miRNAs leads to well differentiation and better prognosis.

**Fig 9:** Schematic model showing the role of NF-κB and miRNA in oral cancer stem like cells (OCSCs) and their modulation in presence or absence of HPV16 infection and their interaction with other gene products leading to either good or worst prognosis when treated. (Thickness of arrow and size of each NF-κB protein has been drawn proportionately).

## Methods

### Cell lines and cell culture

The present study has been carried out using three cell lines, one HPV-16 positive OSCC cell line, UD-SCC-2 (gift from Dr. Henning Bier, University of Dusseldorf, Germany) and two HPV-negative OSCC cell lines, UPCI:SCC131 and UPCI:SCC84 (kind gift from Dr. Susanne M. Gollin, University of Pittsburgh, Pittsburgh, PA, USA and Prof. Arun Kumar, Indian Institute of Science, Banglore, India. The UD-SCC2 cell line was grown in RPMI 1640 medium while UPCI: SCC131 and UPCI: SCC84 cells were grown in DMEM medium (Sigma Aldrich) supplemented with 10% Foetal bovine serum (FBS), 1% Penicillin and Streptomycin (Gibco, Thermo Fisher Scientific Inc., MA USA) at 37°C in a humidified atmosphere containing 5% CO_2_.

### Collection of tumor specimens, HPV detection and establishment of primary culture

A total of 12 oral tumor tissue specimens were collected from ENT department of Sir Ganga Ram Hospital, New Delhi, India. Written informed consent was obtained from all the subjects prior to their inclusion in the study. The study was carried out as per the institutional ethical guidelines and approval from Institutional Ethics Committee of Dr. B.R. Ambedkar Center for Biomedical Research (ACBR), University of Delhi, Delhi, India (ACBR/09/13/IHEC/73) and Sir Ganga Ram Hospital, New Delhi (EC/03/16/896), registered with the Drug Controller General of India (DCGI), Government of India. The HPV diagnosis of oral cancer biopsies were done by standard protocol being followed in our lab [75]. The histopathological diagnosis and tumor staging was done by the experienced pathologist from Sir Ganga Ram Hospital. The study was carried out in accordance with the guidelines and principles of the Helsinki Declaration. Primary cultures of oral tumor tissues were established which were collected in dissociated balanced salt solution (DBSS) containing antibacterial/antimycotic agents as described by Turin and colleagues [76]. The purified primary cultures were used for side population analysis for isolation of oral cancer stem cells.

### Isolation of CSCs from oral cancer cell lines and primary tumor cultures by side population (SP) analysis

SP analysis was based on the previously described method with slight modifications [77]. Briefly, cells from primary culture or cell lines were incubated (1X10^6^ cells/ml) in pre-warmed DMEM supplemented with 2% Fetal Bovine Serum (Sigma) and 10 mM HEPES (Sigma) containing 5 μg/ml Hoechst 33342 at 37°C in a water-bath for 90 minutes with intermittent mixing. The control cells were incubated either alone or in the presence of 50 μM Verapamil (Sigma). After incubation, stained cells were washed and re-suspended in ice-cold HBSS (Sigma) supplemented with 2% FBS. Propidium iodide (1 μg/ml) (sigma) was added immediately before analysis to label dead cells, which were excluded from the analysis. Analysis and sorting was performed on FACS Aria III (BD Biosciences) using Diva Software. The Hoechst 33342 dye was excited with UV laser at 355 nm and emission was collected using 450/50 nm and 675LP filters that allow detection of Hoechst blue and red. Briefly, after completion of staining debris were excluded from cells on the basis of forward scatter (FSC) and side scatter (SSC) on flow cytometer. In order to confirm that signal is arising from single cells, cell doublets and aggregates were gated out based on SSC area (SSC-A) versus height (SSC-H) properties of cells. Dot plot is drawn on a linear scale in presence or absence of Verapamil. SP cells are recognized as a dim tail extending first on the left side of G0/G1 cells towards the lower ‘‘Hoechst Blue” signal. SP cells were gated later on the limit of Hoechstdim staining during Verapamil inhibition included fewer SP cells recognized as a dim tail extending from main population with a characteristic low fluorescence, whereas intense fluorescence signals of bulk population were defined as NSP cells [78].

### Sphere formation assay

For sphere formation, FACS sorted SP and NSP cells from primary tumor culture and cell lines were seeded at density of 1X10^4^ cells on 6- well plates (corning) precoated with 1.2% Poly-HEMA (sigma) in serum free DMEM-F12 medium (Gibco) supplemented with 10ng/ml basic fibroblast growth factor, 10 ng/ml epidermal growth factor and B27 (Invitrogen) or defined serum free medium (DSFM) for 7–10 days. Sphere forming efficiency (SFE) was calculated using the procedure described earlier [39]. Primary spheres were dissociated mechanically and enzymatically using Accutase (Gibco, life technologies) to break up sphere clusters and generate single cell suspension, counted and re-seeded to generate secondary and tertiary spheres in1.2% Poly-HEMA precoated 6-well plates [40]. SP cells from primary culture or cell lines were enriched first as spheres in ultra low adherence condition and then spheres were pooled for carrying out experiments.

### Flow cytometric characterization of CSCs

For further characterization of CSC phenotype of sphere forming SP cells, flow cytometry was used. Spheres were enzymatically dissociated into single cell suspension (1X10^6^). Cells were washed twice with PBS and were stained with CD133-PE and CD117-APC (550412; BD Pharmingen) for 45 minutes at 4°C. Respective mouse IgG isotype were used as control. After incubation cells were washed with PBS and stained with fluorochrome conjugated anti mouse IgG Alexa Fluor 546 (invitrogen) at a dilution of 5 μl of antibody per 10^6^ cell and re incubated further in dark on ice for 30 minute, washed, re-suspended in HBSS and stained by Propidium iodide (1 μg/ml). Analysis and sorting were performed on FACS Aria II using Diva Software.

### Protein extraction and Western blotting

Nuclear extracts from SP, NSP, Parental cells from cell lines and primary tumor culture were prepared by the method of Dignam [79] with minor modifications [6]. Standard Bradford method (Bio-Rad laboratories, Inc. CA) was used to determine the concentration of nuclear protein extracts spectrophotometrically and proteins were stored at − 80 °C till further use. Whole cellular protein/Nuclear protein was separated by electrophoresis on 12/10% SDS–PAGE for expression analysis of CSC markers and NF-κB family proteins respectively and transferred to PVDF membrane. The primary antibodies used were: β- actin (C-11), Oct-3/4 (sc-5279), HCAM (sc-7297), SOX2 (sc-17320), p50 (sc-114), p65 (sc-109), p52 (sc-298), c-Rel (sc-70) and RelB (sc-226) (Santa Cruz Biotechnology, USA) in TBST buffer containing 3% nonfat milk at 4°C overnight and subsequently with anti-mouse and rabbit anti-goat secondary antibody conjugated with peroxidase (Santa Cruz) at 4°C for 3 hour. The immunoblots were visualized by Luminol detection kit and membrane was reprobed for β-actin expression as an internal control [75]. The ratio of the specific proteins to β-actin was calculated. The quantitative densitometric analysis was performed using Image J software.

### Electrophoretic mobility shift assay (EMSA)

Electrophoretic mobility shift assay (EMSA) was performed to detect the NF-κB DNA- binding activity in the nuclear extracts, as described earlier [6, 14] using the following oligonucleotides: NF-κB consensus sequence 5’-AGT TGA GGG GAC TTT CCC AGGG C-3’ (consensus binding sites are underlined), Oct-1 5’-TGT CGA ATG CAA ATC ACT AGA A-3’. The oligos were synthesized from Promega IDT DNA synthesizer using phosphoramitide chemistry. EMSA was carried out either with γ32P-labeled double stranded oligos or 5’ Cy3 labeled oligonucleotides. These oligos were annealed. Briefly, a binding reaction of 10μg nuclear extract with 10pmoles of Cy3 labeled double-stranded oligonucleotides was performed in a 25μl reaction volume containing 50% Glycerol, 60 mM HEPES pH 7.9, 20 mM Tris-HCl pH 7.9, 300 mM KCl, 5 mM EDTA, 5 mM DTT, 100 μg/ml of bovine serum albumin, 2.5 μg of poly (dI-dC) for 30 min at room temperature. The DNA–protein complexes were resolved on 6% non-denaturing polyacrylamide gel (29:1 cross-linking ratio) gel in 0.5X Trisborate- EDTA (TBE) buffer or in buffer containing 89mM Tris, 89mM boric acid (pH 7.5), at 10V/cm at 6°C [80]. The gel was scanned on Typhoon phosphoimager (GE Biosciences).

Binding specificity was confirmed by pre-incubation with a 100-fold molar excess of homologous unlabelled oligonucleotide of NF-κB and heterologous consensus sequence of the Oct-1 transcription factor. For monitoring composition of NF-κB complex by supershift assay, 2 μg of polyclonal antibodies (Abs) directed against each NF-κB family member (Santa Cruz, USA) were added and the reaction mixture was further incubated for 1 hour at 4°C. The rabbit polyclonal antibodies against following NF-κB proteins were used: NF-κB: p50, p65, p52, c-Rel and RelB. The quantitative densitometric analysis was performed using Image J software.

### RNA extraction

The total RNA was extracted from Parental, SP, NSP cells from all three cell lines using mirVana^™^ miRNA isolation kit (Ambion, USA) according to manufacturer’s protocol using 1X10^6^ cells. RNA concentration and purity were determined by using Nanodrop ND-1000.

### Quantitative real-time PCR

#### cDNA synthesis

For miRNA expression analysis, cDNA was synthesized from RNA extracted from Parental, sorted SP and sorted NSP cells of cell lines using specific miRNA RT primers of Taq-Man MicroRNA Reverse Transcription kit (Applied Biosytem, USA). For cDNA preparation, 10 ng of total RNA per 15-μL RT reaction were used. For HPV-16 E6 and E7 gene expression analysis, cDNA was prepared from HPV16+ve UD SCC2 cell line and HPV+ve patient biopsies from RevertAid first strand cDNA synthesis kit (Thermoscientific) as per manufacturer’s protocol.

#### Real-time PCR

Real-Time PCR was performed using the TaqMan universal mastermix kit/SYBER green master mix (Applied Biosystem, USA) as described previously [40, 81]. Real-Time PCR for miRNA expression analysis was carried out using primers hsa-miR-21, hsa-miR-34a, hsa-miR-155 and RNU6B as a reference control while primers E6, E7 and β globin as housekeeping gene were used for HPV16+ve E6/E7 gene expression (Primer sets are listed in S2 Table). The fold change was calculated based on the threshold cycle (CT) value using the following formula: Relative Quantification (RQ) = 2−ΔΔCT. All experiments were run in triplicate.

### Statistical analysis

The data analysis was performed using the statistical software Graph Pad Prism (version 6.0) and image J software.To detect the difference in the miRNA expression level between parental, SP and NSP cells was done using the Two-Way ANOVA test followed by Bonferroni post hoc test for significant difference. The expression profile of NF-κB proteins and CSC markers was determined using Fischer’s exact test and student t-test (two tailed). Data were presented as means±SE of three or more independent experiments. The difference was considered statistically significant when P< 0.05.

### Ethics approval and consent to participate

The study was ethically approved by the Institutional Ethics committee of Dr. B. R. Ambedkar Center for Biomedical Research, University of Delhi, India and Sir Ganga Ram Hospital (New Delhi, India.

## Supporting information

S1 Fig FACS analysis data of Flow cytometric (FACS) analysis of SP cells in OSCC cell lines. (PDF)

S2 Fig Flow cytometric (FACS) analysis of SP cells in OSCC cell lines. (TIF)

S3 Fig FACS analysis data of functional characterization of SP cells present in OSCC cell lines. (PDF)

S4 Fig Constitutive activation and DNA binding activity of NF-κB in HPV+ve and HPV-ve oral cancer cells. (TIF)

S5 Fig Relative expression level of selected miRNAs in SP, NSP and their parental controls from UD-SCC2 (HPV16+ve), UPCI:SCC131 (HPV-ve) and UPCI: SCC 084 (HPV-ve). (TIF)

S1 Table The original raw data of microRNA expression in OSCC cell lines. (XLS)

S2 Table Primer sequences used for expression analysis of HPV-16 viral oncogenes E6 and E7. (DOC)

## Abbreviations

CSCs: Cancer stem cells
CT: threshold cycle
FACS: Fluorescence Activated Cell Sorter
HNSCC: Head and neck squamous cell carcinomas
HR-HPV: High risk human papilloma virus
miRNA or miR: microRNA
NF-kB: Nuclear factor kappa B
NSP: Non-side population
OCSCs: Oral Cancer Stem like cell
OSCC: Oral squamous cell carcinoma
RQ: Relative Quantification
SP: Side population
